The article "Identification of Key Genes and Pathways for Enchondromas by Bioinformatics Analysis" was retracted in 2024. Reasons: signs of a paper mill; concerns about the results or conclusions; concerns about the authorship; concerns about a third party's involvement.

# Identification of Key Genes and Pathways for Enchondromas by Bioinformatics Analysis

**DOI:** 10.1177/1559325820907536

**Published:** 2020-03-30

**Authors:** Tianlong Wu, Honghai Cao, Lei Liu, Kan Peng

**Affiliations:** 1 Department of Sports Medicine, The First Bethune hospital of Jilin University, Changchun, Jilin, China; 2 The Chinese PLA General Hospital, Beijing, China; 3 Department of Pain, Qianfoshan Hospital Affiliated to Shandong University, Jinan, Shandong, China; 4 Department of Joint Surgery, Xi’an Hong Hui Hospital, Xi’an Jiaotong University Health Science Center, Xi’an, Shaanxi, China

**Keywords:** gene ontology, enchondromas, biomarkers

## Abstract

**Background:**

The risk of malignant transformation of enchondromas (EC) toward central chondrosarcoma is increased up to 35%, while the exact etiology of EC is unknown. The purpose of this research was to authenticate gene signatures during EC and reveal their potential mechanisms in occurrence and development of EC.

**Methods:**

The gene expression profiles was acquired from Gene Expression Omnibus database (no. GSE22855). The gene ontology (GO), protein–protein interaction (PPI) network and Kyoto Encyclopedia of Genes and Genomes pathway (KEGG) enrichment analyses were utilized to identify differentially expressed genes (DEGs).

**Results:**

Finally, 242 DEGs were appraisal, containing 200 overregulated genes and 42 downregulated genes. The outcomes of GO analysis indicated that upregulated DEGs were mainly enriched in several biological processes containing response to hypoxia, calcium ion, and negative regulation extrinsic apoptotic signaling pathway. Furthermore, the upregulated DEGs were enriched in extracellular matrix (ECM)–receptor interaction, protein processing in endoplasmic reticulum and ribosome, which was analyzed by KEGG pathway. From the PPI network, the top 10 hub genes were identified, which were related to significant pathways containing ribosome, protein processing in endoplasmic reticulum, and ECM-receptor interaction.

**Conclusion:**

In conclusion, the present study may be helpful for understanding the diagnostic biomarkers of EC.

## Introduction

Originated from hyaline cartilage, chondroma is called enchondromas (EC) when it appears in medullary cavity. Enchondroma is more common in men and its peak incidence is at 20 to 30 years old. In any area of the moving spine, these cancers may happen.^1^ The exact etiology of EC is unknown. If hemangiomas are also existing, multiple EC or “Enchondromatosis” is called Ollier or Maffucci syndrome. The risk of malignant transformation of EC toward central chondrosarcoma, which is a malignant bone tumor forming hyaline cartilage and arising centrally in the medullary cavity of bone,^2-4^ is increased up to 35%. Therefore, comprehending the molecular mechanisms associated with the pathological process of EC is critical for developing more valid diagnostic and therapeutic strategies.

High-throughput platforms for analyzing gene expression, such as microarrays, are gaining increasing attention and are promising tools for medical oncology with a wide range of clinical applications, such as diagnosis, prognosis prediction, discovery of potential therapeutic targets, and so on.^5^ At present, researchers utilize microarray technology combined with bioinformatics to analyze the expression changes of mRNA in the occurrence and development of EC.^2^

In this study, we obtained the original data from Gene Expression Omnibus (GEO) database, which is repository for microarray data deposit and retrieval. To identify differentially expressed genes (DEGs), we compared the gene expression profiles of tumor cells in EC patients and normal tissues. Whereafter, the DEGs were filtrated by gene ontology (GO) and pathway enrichment analysis. These results might offer a theoretical basis for ulterior exploration of diagnostics, prognosis, and drug targets for EC.

## Methods

### Microarray Data

This research has been approved by the institutional review board of the authors’ affiliated institutions. The gene expression profiles was obtained from GEO (http://www.ncbi.nlm.nih.gov/geo/) database (no. GSE22855). GSE22855, which was established on the platform of Illumina Beadarray v3.0 (Illumina Inc, San Diego, California), was submitted by Pansuriya. There were 13 samples in this data set, including 7 EC samples and 6 normal samples (growth plate and cartilage).

### Identification of DEGs

Seven EC samples and 6 normal samples were analyzed with GEO online analysis tool GEO2R (https://www.ncbi.nlm.nih.gov/geo/geo 2 r/). Only genes with an adjusted *P* < .05 and |log_2_ fold change (FC)| ≥1 were choiced as DEGs.

### Gene Ontology and Kyoto Encyclopedia of Genes and Genomes Pathway (KEGG) Analysis of DEGs

Gene ontology collects structured, defined, and controlled vocabulary for massive genes annotation, which is a diffusely utilized method for biology.^6^ Kyoto Encyclopedia of Genes and Genomes (http://www.genome.jp/) database integrates the information for genome, chemistry, and function and is also one of the most commonly used bioinformatics databases in the world.^7^ Visualization and Integrated Discovery (DAVID) can quickly, systematically, and comprehensively annotate the functions of various of genes and enrich and analyze the genes and calculate the enrichment fraction. DAVID also provides a fast conversion function between gene names.^8,9^ The screened DEGs, which were analyzed by GO enrichment and KEGG pathway, were carried out utilizing DAVID online tool (https://david.ncifcrf.gov/). *P* < .05 was considered as significant.

### Integration of Protein–Protein Interaction Network

To evaluate the protein–protein interaction (PPI) information, the online tool Search Tool for the Retrieval of Interacting Genes (STRING) database is used.^10^ From 1133 organisms, STRING (version 9.0) contains 5 214 234 proteins. To assess the interaction among DEGs, the DEGs were mapped to STRING, and only the combined score >0.4 were chosen as significant. The Cytoscape software (version 3.6.1) was employed to construct PPI networks.^11^

## Results

### Identification of DEGs

Based on GEO2R analysis, a total of 242 DEGs (200 upregulated genes and 42 downregulated genes) were identified based on *P* < .05 and fold change (FC) ≥2.0 criteria. Vocano plot and heat map of DEGs are shown in Figures 1 and 2. The top 10 significant upregulated and top 10 significant downregulated DEGs are illustrated in Table 1.

**Figure 1.** Vocano plot of differentially expressed genes (DEGs). Red: upregulated genes; Green: downregulated genes.

**Figure 2.** Heat map of TOP100 differentially expressed genes (DEGs). Red: upregulation; Blue: downregulation.

**Table 1.** The Top10 Significant Upregulated and Downregulated DEGs Involved in EC.

Regulated	Row Names (tT)	logFC	*P* Value
upregulated	PENK	6.282102002	6.88E-09
	FOSB	4.577903408	3.76E-05
	TRIB3	3.0873647	1.56E-06
	DLK1	2.822339106	2.532203E-03
	THBS3	2.781973194	1.71E-06
	DSPG3	2.748504195	2.167939E-03
	SLC27A2	2.7150976	7.26E-07
	NELL1	2.6088895	2.56E-07
	PRSS23	2.405676176	3.55E-06
	C1orf24	2.399071104	1.84E-05
downregulated	ECRG4	−5.69745338	2.76E-06
	LOXL4	−4.377491179	9.47E-07
	SERPINA5	−2.897102353	9.32E-07
	DDIT4	−2.747095868	2.392049E-03
	GBP2	−2.441809126	1.82214E-04
	TF	−2.367202109	1.06E-05
	ADM	−2.222022278	2.072312E-03
	FAM46C	−2.201757972	9.41559E-4
	ERRFI1	−2.197346735	7.16472E-4
	MT1G	−2.192670709	3.868122E-3

Abbreviations: DEG, differentially expressed gene; EC, enchondroma.

### Gene Ontology Term Enrichment Analysis

The results of GO analysis displayed that DEGs were obviously enriched in biological processes containing response to hypoxia, response to calcium ion, negative regulation of extrinsic apoptotic signaling pathway, axon extension involved in axon guidance, collagen fibril organization, interleukin-1-mediated signaling pathway, and so on (Figure 3). For molecular function, the DEGs were enriched in extracellular matrix (ECM) structural constituent, integrin binding, structural constituent of ribosome, heparin binding, kinase activity, receptor binding, and so on (Figure 3). In addition, the DEGs were distinctly enriched in cytosolic ribosomal subunit, ribosome and basement membrane, endoplasmic reticulum (ER) lumen, proteinaceous ECM, and ECM, and so on, which were analyzed by GO cell component (Figure 3). The relationship between the DEGs and GO terms, as well as the logFC of the DEGs are shown in Figure 4.

**Figure 3.** Gene ontology (GO) enrichment analysis.

**Figure 4.** Gene ontology (GO) Chord.

### Kyoto Encyclopedia of Genes and Genomes Pathway Analysis

Analyzing by KEGG analysis, the most visibly enriched pathways of the upregulated and downregulated DEGs are presented Table 2 and Figure 5. The upregulated DEGs were enriched in ECM-receptor interaction, protein processing in ER, ribosome, focal adhesion, and PI3K-Akt signaling pathways, while the downregulated DEGs were enriched in mineral absorption pathway.

**Table 2.** Enriched Pathways of DEGs.

Term	Count	*P* Value	Genes
Ribosome	10	6.22E-05	RPS28, RPL23, RPL14, RPL7, RPS3A, RPL21, RPLP1, RPS15A, RPL5, RPL7A
ECM-receptor interaction	7	8.95E-04	COL4A2, TNC, COL3A1, THBS1, COL11A2, COL11A1, THBS3
Protein processing in endoplasmic reticulum	9	1.528426E-03	ATF4, SEC61B, HSPA1A, RPN2, MAN1A1, DDOST, SAR1A, UBE2E2, RBX1
Focal adhesion	9	5.197548E-03	COL4A2, CAV1, TNC, COL3A1, PDGFD, THBS1, COL11A2, COL11A1, THBS3
PI3K-Akt signaling pathway	11	1.3784745E-02	COL4A2, ATF4, TNC, COL3A1, CDK6, PDGFD, THBS1, COL11A2, COL11A1, THBS3, DDIT4
Mineral absorption	4	2.1672904E-02	SLC11A2, TF, FTH1, MT1G

Abbreviations: DEG, differentially expressed gene; ECM, extracellular matrix.

**Figure 5.** Kyoto Encyclopedia of Genes and Genomes (KEGG) pathway enrichment analysis. Red: upregulated genes; Green: downregulated genes.

### Protein–Protein Interaction Network

As displayed in Figure 6, the PPI network was constructed based on the information of the STRING database. Besides, with higher degrees, the top 10 hub nodes were identified. These hub genes included protein transport protein Sec61 subunit beta (SEC61B), ribophorin II (RPN2), glycosyltransferase 48 kDa subunit (DDOST), 40S ribosomal protein S15 (RPS15A), 60S ribosomal protein L23 (RPL23), 60S ribosomal protein L7a (RPL7A), 60S acidic ribosomal protein P1 (RPLP1), 40S ribosomal protein S3a (RPS3A), 60S ribosomal protein L14 (RPL14), and 40S ribosomal protein S28 (RPS28). Utilizing MCODE plugin, a total of 201 nodes and 271 edges were obtained. The top 3 significant modules are shown in Figure 7. Enrichment analysis displayed that the genes in module 1-3 were chiefly concerned with ribosome, protein processing in ER, ECM-receptor interaction, and protein digestion and absorption pathways (Tables 3 [Table table4-1559325820907536]-5).

**Figure 6.** Protein–protein interaction network of differentially expressed genes (DEGs). Circles represent genes, lines represent the interaction of proteins between genes, and the outcomes within the circle represent protein structures. Line color represents protein interactions.

**Figure 7.** Top 3 modules from the protein–protein interaction network. A, module 1; B, module 2; C, module 3.

**Table 3.** Respective Enriched Pathways of Module 1.

Term	Count	*P* Value	Genes
hsa03010: Ribosome	10	7.12E-14	RPS28, RPL23, RPL14, RPL7, RPS3A, RPL21, RPLP1, RPS15A, RPL5, RPL7A
hsa04141: Protein processing in endoplasmic reticulum	3	0.033412617	SEC61B, RPN2, DDOST

**Table 4. table4-1559325820907536:** Respective Enriched Pathways of Module 2.

Term	Count	*P* Value	Genes
hsa04512: ECM-receptor interaction	3	1.57E-04	COL4A2, COL3A1, COL11A1
hsa04974: Protein digestion and absorption	3	1.60E-04	COL4A2, COL3A1, COL11A1
hsa05146: Amoebiasis	3	2.33E-04	COL4A2, COL3A1, COL11A1
hsa04510: Focal adhesion	3	8.85E-04	COL4A2, COL3A1, COL11A1
hsa04151: PI3K-Akt signaling pathway	3	0.002485904	COL4A2, COL3A1, COL11A1
hsa04611: Platelet activation	2	0.037275359	COL3A1, COL11A1

Abbreviation: ECM, extracellular matrix.

**Table 5.** Respective Enriched Pathways of Module 3.

Term	Count	*P* Value	Genes
hsa04120: Ubiquitin mediated proteolysis	4	7.63E-06	CBLB, SOCS3, UBE2E2, RBX1

## Discussion

In this article, utilizing bioinformatics analysis, 200 overexpressed and 42 downregulated DEGs were identified. Following that, GO and KEGG pathway analyses were performed to further understand the interactions of DEGs. Microarrays and high-throughput sequencing have been diffusely utilized to forecast potential therapeutic targets for cancers, because they can offer thousands of genes expression levels in the human genome. The consequences of GO term analysis demonstrated that upregulated DEGs were chiefly related to response to hypoxia, response to calcium ion, and negative regulation of extrinsic apoptotic signaling pathway. Ca^2+^ modulates numerous aspects of tumors, containing growth, migration, apoptosis, angiogenesis, and so on.^12^ Studies have demonstrated that Ca^2+^ signaling was remodeled in various tumors, including the changes of expression levels or activities of Ca^2+^ transporters and channels.^13-15^ Infinite growth of tumor cells is the result of inhibition of tumor cell apoptosis; therefore, apoptosis obstacles, including negative regulation of extrinsic apoptotic signaling pathway, may have a close relationship with the occurrence and development of tumors.^16^ One of the most crucial characters for solid cancers is anoxic microenvironment. Besides, one of the prerequisites for cancer metastasis is that cancer cells can accelerate the formation of unnormal blood vessels by secreting a variety of vascular growth factors, which occur under anoxic conditions.^17^

Moreover, the enriched KEGG pathways in the upregulated DEGs contained ECM-receptor interaction, protein processing in ER, ribosome, focal adhesion, and PI3K-Akt signaling pathways, while the downregulated DEGs were enriched in mineral absorption pathway. Extracellular matrix-receptor interaction is the pathway involved in lung adenocarcinoma, gastric cancer, and so on.^18,19^ As reported, the increased activation of unfolded protein responses mediators in the ER in different tumor types patients and their upregulation usually related to poor prognosis and resistibility to many kinds of treatments.^20^ Mechanistic data have indicated that ribosome biosynthesis disorders have a broader effect in most spontaneous cancers progression and development.^21^ The PI3K-Akt pathway is one of the most commonly dysregulated pathways in tumors.^22,23^ Some reports have demonstrated that abnormal absorption of mineral ions including Ca^2+^ and Zn^2+^ is closely associated with the occurrence and development of tumor.^24^

We also structured the PPI network with DEGs and showed 10 top degree hub genes: SEC61B, RPN2, DDOST, RPS15A, RPL23, RPL7A, RPLP1, RPS3A, RPL14, and RPS28. Fan et al^25^ reported that transport protein Sec61 subunit beta (SEC61β) was expressed high in human colorectal cancer, detection of SEC61β autoantibody levels might offer a selective testing pointer for CRC, especially among patients in early stage. Ribophorin II (RPN2), mediates CD63 glycosylation and as a portion of an N-oligosaccharyl transferase complex, can regulate drug resistance and invasion in breast cancer, cancer malignancy, and MDR1 localization.^26^ It has been reported that RPN2 correlates with a variety of malignant cancers, such as colorectal cancer,^27^ breast cancer,^28^ and so on. RPN2, as a hopeful prognostic indicator in human gastric adenocarcinoma, is a valid biomarker to forecast the consequence of chemotherapy for terminal gastric cancer,^29^ Zhang et al^30^ reported that DDOST was one of the core genes involved in bladder cancer. Ribosomes have a complicated structure and functions, which are important sites for proteins synthesis associated with expression and transmission of genetic information in human. Ribosomal proteins act a momentous influence on human diseases, containing the origination and evolution of malignancies.^31^

## Conclusion

In conclusion, through bioinformatics analysis, our work identified some pivotal DEGs and cellular pathways concerned with EC occurrence and development, which might offer a basis for EC treatment. Nevertheless, ulterior experimental studies should be executed to affirm the expression and function of the identified genes in protein level, which will be reported in future articles.
